# Chemotherapy with a TP Regimen in Combination with Stereotactic Radiotherapy Could Significantly Optimize the Clinical Efficacy of NSCLC Treatment

**DOI:** 10.1155/2022/8495452

**Published:** 2022-06-14

**Authors:** Chenglin Wu, Biyu Chen, Meifang Wang, Yijun Tang

**Affiliations:** Department of Respiratory and Critical Care Medicine, Shiyan Taihe Hospital, Shiyan 442000, Hubei, China

## Abstract

The changes in lifestyle and bad living habits have a significant impact on the health of people, resulting in an increasing prevalence of lung cancer. The most prevalent kind of lung cancer is nonsmall cell lung cancer (NSCLC), which accounts for around 80% of all cases. Chemotherapy is a common treatment method in clinical practice with certain negative effects. The primary goal of this study is to investigate the clinical efficacy of stereotactic radiotherapy in combination with a docetaxel plus cisplatin (TP) chemotherapy regimen in patients with nonsmall cell lung cancer (NSCLC) and their impact on the levels of cytokeratin fragment 21-1 (CYFRA21-1) and metastasis-associated lung adenocarcinoma transcript 1 (MALAT1) in NSCLC patients. Eighty patients who were admitted to the hospital between November 2016 and November 2019 were recruited and assigned to receive either chemotherapy with a TP regimen (the control group) or chemotherapy with a TP regimen plus stereotactic radiotherapy (the observation group). The WHO response evaluation criteria (REC) for solid tumors were adopted to analyze short-term efficacy, and the Karnofsky performance status (KPS) score was used to assess the quality of life by recording adverse reactions in the blood system, kidney, gastrointestinal tract, bladder, nervous system, and heart. The levels of CYFRA21-1 and MALAT1 in serum before and after the treatment were determined and compared. As a result, the observation group showed higher total efficacy and MALAT1 level, better quality of life, and lower CYFRA21-1 level than the control group (*P* < 0.05). Stereotactic radiotherapy plus TP regimen chemotherapy resulted in significantly better progression-free survival, overall survival, survival rate, and long-term prognosis versus chemotherapy alone. Moreover, combined therapy was associated with a lower incidence of hemoglobin reduction, gastrointestinal reaction, and renal impairment versus TP regimen chemotherapy (*P* < 0.05). Therefore, we concluded that stereotactic radiotherapy plus chemotherapy with a TP regimen significantly optimizes the clinical efficacy of the NSCLC treatment.

## 1. Introduction

Lung cancer is a common clinical malignant tumor in the respiratory system, with a high incidence and mortality [1]. NSCLC accounts for about 80% of all lung cancer cases [2]. Due to the insidiousness of symptoms in the early stage, NSCLC usually progresses to an advanced stage by the time of diagnosis, where patients are mostly inoperable, resulting in a somber prognosis and a lower five-year survival rate [3]. Therefore, effective disease control is the key to the treatment of advanced NSCLC.

Chemotherapy is a commonly used treatment in clinical practice but has severe toxic and side effects that impair the immune function of the body and compromise the quality of life [4]. Therefore, it is of great significance to explore treatments with an excellent tumor-killing effect and small toxic side effects for improving the patients' life quality. Stereotactic radiation is initially used to treat extracranial malignancies and is now commonly used to treat inoperable early stage NSCLCs. Moreover, stereotactic radiotherapy is as effective as surgical treatment for patients with high surgical risks [5]. Cytokeratin 21-1 fragment (CYFRA21-1) is currently an important clinical marker for the diagnosis of NSCLC [6]. Research has revealed that the serum level of CYFRA21-1 could reflect the patients' quality of life and indicate the risk of recurrence. MALAT1 is a member of the long-chain noncoding RNA family and possesses transcriptional and epigenetic regulatory effects. It has been reported that MALAT1 is abnormally expressed in tumor tissues and exerts an essential regulatory effect on the radiosensitivity of NSCLC [7].

Stereotactic radiotherapy concentrates X-rays or radiation beams to a point from all directions to produce a high dose of the radiation effect on the tumor, with a minimal radiation dose to the surrounding normal tissues. In addition, stereotactic radiotherapy is accurate in positioning, with simple operation and high safety, and has been mostly used for intracranial tumor treatment in the past.

The main contributions of this study are as follows. (1) We investigated the clinical efficacy of stereotactic radiotherapy in combination with a docetaxel plus cisplatin (TP) chemotherapy regimen in patients with NSCLC and their effects on the levels of CYFRA21-1 and NSCLC patients. (2) The changes in serum CYFRA21-1 and MALAT1 levels before and after treatment have been observed and analyzed. The aim of this study was to explore the clinical application value of stereotactic radiotherapy plus TP regimen chemotherapy to provide a reference for the clinical treatment of NSCLC. (3) The results illustrate that the proposed protocol is better than conventional methods in terms of clinical efficacy.

The rest of the study is organized as follows.  Section 2 describes the details of the participants and methods in this study.  Section 3 shows the results of the present study. A comprehensive discussion is presented in Section 4. Finally, Section 5 summarizes the results of this study.

## 2. Patients and Methods

This section includes the information about patients recruited in this study and the methods of the experiments.

### 2.1. General Information

With the approval of the Ethics Committee of Shiyan Taihe Hospital, No. TH29-19, 80 patients admitted to this hospital between November 2016 and November 2019 were randomly recruited and assigned to an observation group or a control group. In the observation group, there were 27 males and 13 females, with a mean age of (48.37 ± 3.84) years, 26 cases of tumor stage III and 14 cases of stage IV, a mean KPS score of (70.28 ± 3.43) points, and 29 cases with a history of smoking. In the control group, there were 25 males and 15 females, with a mean age of (48.64 ± 3.93) years, 25 cases of tumor stage III and 15 cases of tumor stage IV, a mean KPS score of (70.35 ± 3.65) points, and 28 cases with a history of smoking. The baseline patient profiles of the two groups were comparable (*P* > 0.05).

### 2.2. Inclusion Criteria

The following steps specify the inclusion criteria for the patients with NSCLS in this research study.

1. Confirmed diagnosis of stage III or IV NSCLC through pathological biopsy, bronchoscopy, imaging examination, and surgical histopathological examination
2. Patients with complete imaging data
3. Patients with regular follow-up and treatment intervention
4. Patients with a functional status score of ≥60 points
5. Patients and family members provided written informed consent

### 2.3. Exclusion Criteria

Exclusion criteria are specified on the basis of the following steps.

1. Patients with severe liver and kidney disease problems
2. Patients with mental diseases or consciousness disorders
3. Patients with chemotherapy tolerance of <2 weeks
4. Patients with organ dysfunctions
5. Patients with other antitumor regimens
6. Patients with withdrawal of consent

### 2.4. Methodology

Patients in the control group received chemotherapy with a TP regimen, and patients in the observation group received chemotherapy with a TP regimen plus stereotactic radiotherapy.

In the control group, patients were intravenously injected with paclitaxel 135 mg/m^2^ on day 1 and cisplatin 25 mg/m^2^ from day 1 to day 3. A similar chemotherapy protocol was introduced to patients in the observation group. Patients in the observation group additionally received stereotactic radiation. Patients, in a supine position, lifted their hands on top of their heads and fixed by vacuum phantom, breathed quietly, and were scanned by a thin-layer spiral CT with the thickness of 5 mm. CT scan images were imparted into the system to design and optimize the three-dimensional treatment protocol. The patient's body surface, vital tissues, and organs were outlined, the clinical target volume was 5 mm outside the gross tumor volume (GTV), and the planning target volume (PTV) was 5–8 mm of the clinical target area. Using the fixed field technique, 5–7 radiation fields were selected, and the geometric center of PTV was determined by the radiographic design to ensure that the target area avoided important organs and was included in the target field. The evaluation was performed using isodose curve synthesis and dose-volume histogram to determine the best treatment plan for the patient. The lungs were irradiated with less than 25% of the total lung volume of 20 Gy, and the maximum irradiated doses were ≤45 Gy, 60 Gy, and 35 Gy for the spinal cord, esophagus, and heart, respectively. The stereotactic radiotherapy treatment plan was transmitted to a network computer, and the patient's lung lesions, ipsilateral hilum, and integrated lymphatic drainage areas were irradiated with 2.5–4.85 Gy per time, 5 times a week for a total of 10–12 times.

Due to the serious adverse reactions of NSCLC patients during radiotherapy and chemotherapy, our hospital attempted to alleviate the adverse reactions of patients and improve the clinical treatment by treating the patients with Qudu Fuzheng decoction, which consists of Coicis Semen 30 g, Astragali Radix 30 g, Poria 30 g, Pseudostellariae Radix 20 g, Herba Hedyotis 15 g, Ophiopogonis Radix 15 g, Agrimoniae herba 15 g, Herba Scutellariae Barbatae 15 g, *Euphorbia lunulata* Bunge 15 g, Radix Cat's Eye 15 g, *Gekko swinhonis* Seu japonicus 10 g, Rehmanniae Radix 10 g, Lycii fructus 10 g, Chinese magnolcavine fruit 10 g, Corni fructus 10 g, scorpion 10 g, and centipede 6 g. Reed rhizome, Platycodonis Radix, Atractylodis Macrocephalae Rhizoma, tangerine peel, and Trichosanthis Fructus were added for phlegm-dampness in the lung. Notoginseng Radix, safflower, peach seed, Platycodonis Radix, and Aurantii fructus were added for the stagnation of the lung channels. Rehmanniae Radix, lily, Fritillariae Thunbergii Bulbus, and white peony root were added for deficiency of both qi and yin, and forsythia, Forsythiae fructus, *Chrysanthemum*, Polygonati Odorati Rhizoma, coastal glehnia root, and Trichosanthis fructus were added for yin deficiency and toxic heat. One dose of the above prescription was decocted with water daily to obtain 200 mL of liquid, which was administered orally with half dose in the morning and a half in the evening. The treatment was continued for 2 cycles with 3 weeks as 1 cycle. Currently, it is used as an adjunct to clinical treatment.

### 2.5. Observation Indicators

The WHO response evaluation criteria (REC) [8] were used to assess the short-term efficacy of patients. It includes complete response (CR), partial response (PR), stable disease (SD), and progressive disease (PD), where (CR + PR)/total number × 100% was recorded as total efficacy. The patients' quality of life was assessed using the KPS score [9]. An increase of more than 10 points in the KPS score indicated improved quality of life, an increase of fewer than 10 points indicated stable quality of life, while a decrease in the KPS score indicated compromised quality of life. The sum of the improved rate and stable rate was recorded as the total improvement rate. Adverse reactions in the blood system, kidney, gastrointestinal tract, bladder, nervous system, and heart system of patients were recorded. Fasting venous blood was collected before and after the treatment and centrifuged to obtain serum, and the level of CYFRA21-1 in blood of patients was determined using ELISA. The levels of MALAT1 and *β*-actin in blood of patients were determined using PCR, and the primer sequences are given in Table 1. In addition, the patients were followed-up every month, and the asymptomatic survival period, the total survival period, and the recurrence were observed and recorded to evaluate the long-term prognosis.

### 2.6. Statistical Methods

In this study, SPSS 20.0 was used for data analyses. Count data are expressed as (*n* (%)) and analyzed using the chi-square test. Measurement data are expressed as (mean ± SD) and analyzed using the LSD *t*-test. If *P* < 0.05, the differences are considered statistically significant.

## 3. Results

The results of this study were evaluated in terms of short-term efficacy, quality of life, serum CYFRA21-1 and MALAT1 levels, progression-free survival and overall survival, survival rates, long-term prognosis, and adverse reactions.

### 3.1. Short-Term Efficacy

The TP chemotherapy regimen plus stereotactic radiotherapy was associated with higher efficacy (65%) versus the TP chemotherapy regimen alone (50%) (*P* < 0.05) (Table 2 and Figures 1, 2).

### 3.2. Quality of Life

Patients in the observation group had a higher quality of life after therapy than those in the control group (*P* < 0.05) (Table 3 and Figures 3, 4).

### 3.3. Serum CYFRA21-1 and MALAT1 Levels

Before treatment, the two groups (observation and control) showed no significant difference in the serum CYFRA21-1 and MALAT1 levels (*P* > 0.05). After treatment, a lower CYFRA21-1 level and a higher MALAT1 level were observed in the observation group as compared to the control group (*P* < 0.05) (Table 4).

### 3.4. Progression-Free Survival and Overall Survival Time

The results showed that the progression-free survival and overall survival time in the observation group were (10.28 ± 2.01) months and (12.36 ± 2.52) months, respectively. The progression-free period and overall survival time in the control group were (8.17 ± 1.58) months and (10.24 ± 2.11) months, respectively. The observation group showed significantly longer progression-free survival and overall survival time than the control group (*P* < 0.05) (Table 5).

### 3.5. Survival Rates

The six-month and one-year survival rates in the observation group were 85.00% and 80.00%, respectively, and those in the control group were 75.00% and 55.00%, respectively. Patients in the observation group showed a significantly higher six-month survival rate and a one-year survival rate than those in the control group (*P* < 0.05) (Figure 5 and Table 6).

### 3.6. Long-Term Prognosis

The local recurrence rate and distant metastasis rate in the observation group in one year were 5.00% and 7.50%, respectively, and those of the control group were 22.5% and 25.00%, respectively. Patients receiving TP regimen chemotherapy combined with stereotactic radiotherapy intervention had a lower one-year local recurrence rate and a distant metastasis rate than patients receiving a TP regimen only (*P* < 0.05) (Table 7 and Figure 6).

### 3.7. Adverse Reactions

The observation group had a significantly lower incidence of hemoglobin reduction, gastrointestinal reaction, and renal impairment than the control group (*P* < 0.05). However, there were no significant differences in the incidence of leukopenia and liver function injury between the two groups (*P* > 0.05) (Table 8).

## 4. Discussion

NSCLC is the most common pathological type of lung cancer. Because of the lack of screening measures and insidious early symptoms, most cases have developed to grades III and IV of tumors, where surgical treatment is considered ineffective [8]. Chemotherapy is the mainstay of the advanced NSCLC. However, chemotherapy is usually accompanied by the disorder of the bone marrow hematopoietic system and the immune system which predisposes patients to inflammatory reactions, nausea, vomiting, decreased immunity, and malnutrition, seriously undermining the therapeutic effect [9]. Radiotherapy has the advantage of low toxic effects, side effects, and promising local treatment effects and is frequently used for cancer treatment [10]. Stereotactic radiotherapy is one of the common radiotherapy approaches and has become the main treatment for early stage NSCLC patients who are inoperable [11].

Stereotactic radiotherapy uses a multifield, noncoplanar, or coplanar irradiation scheme through computer technology to effectively ensure high consistency between the tumor target area and the irradiated high dose area, thereby effectively protecting the adjacent normal tissues while irradiating the tumor target area at high doses [12]. In the present study, the observation group showed higher total efficacy, better quality of life, and a lower incidence of hemoglobin reduction, gastrointestinal reactions, and renal impairment than the control group. However, the incidence of leukopenia and liver function impairment in patients between the two groups showed no noteworthy variance. It has been reported that stereotactic radiotherapy has a high clinical value in the treatment of patients with advanced lung cancer. Moreover, it could improve clinical efficacy, which is similar to the results of the present study [13].

CYFRA21-1 is a soluble fragment of an important cytokeratin-19 in the body, which is widely distributed on the surface of normal tissues, such as squamous or stratified epithelium. It is often considered one of the important markers for the diagnosis and differentiation of lung cancer. It has been reported that CYFRA21-1 has a high diagnostic sensitivity for NSCLC after treatment and shows great potential to evaluate the changes in the patient's condition [14]. MALAT1 is a member of an important long-chain noncoding RNA family in the human body. It has been considered a noise gene in previous studies. In recent years, it has been confirmed that abnormal high expression of MALAT1 is seen in the A549 lung adenocarcinoma cell line [15]. MALAT1 effectively participates in the formation and growth of tumor cells, as well as their invasion and migration, and plays a vital role in the epithelial-mesenchymal transition. The results of the present study demonstrated a lower level of CYFRA21-1 and a higher level of MALAT1 after treatment. Furthermore, chemotherapy with a TP regimen plus stereotactic radiotherapy resulted in better progression-free survival, overall survival, survival rate, and the long-term prognosis versus TP regimen chemotherapy alone. According to analysis, for NSCLC patients with stereotactic radiotherapy combined with TP chemotherapy, the three-dimensional reconstruction technology of stereotactic radiotherapy images can be used to accurately analyze the tumor volume of patients and perform a personalized medical intervention, thus significantly ameliorating the treatment efficacy, improving the survival and reducing the recurrence. Stereotactic radiotherapy combined with the TP chemotherapy regimen for treating NSCLC contributes to improving the quantitative volume dose distribution of patients, effectively controlling the irradiated dose and irradiated volume of main organs, elevating the prognosis of patients and the levels of CYFRA21-1 and MALAT1 in blood. In short, stereotactic radiotherapy combined with TP chemotherapy could significantly improve the clinical efficacy of NSCLC treatment and the levels of CYFRA21-1 and MALAT1 in blood of patients.

Nonsmall cell lung cancer belongs to the category of “lung stagnation” in traditional Chinese medicine. In traditional Chinese medicine, the disease is caused by internal deficiency of positive qi, dysfunction of internal organs, and external invasion of evil and toxin, which lead to loss of lung qi and blood circulation, stagnation of qi and blood stasis, dampness, and phlegm. In the formula of Qudu Fuzheng decoction, Coicis Semen detoxifies and disperses nodules, strengthens the spleen, relieves diarrhea, and promotes diuresis. Poria strengthens the spleen and nourishes the heart, diuresis, and dampness. Astragali Radix benefits qi and consolidates the surface, diuresis, and toxicity. Pseudostellariae Radix benefits the qi, strengthens the spleen, and moistens the lungs. Ophiopogonis Radix generates body fluid and thirst, moistens lungs, and stops cough. Agrimoniae Herba detoxifies and tonifies deficiency, astringent, and stops bleeding. Herba Scutellariae Barbatae clears heat and detoxifies and resolves blood stasis and diuresis. *Euphorbia lunulata* Bunge suppresses cough and dispels phlegm, extracts poison, and disperses nodules. Rehmanniae Radix tonifies blood and nourishes yin. Lycii fructus nourishes the liver and the kidney and moistens the lung. Chinese magnolcavine fruit tonifies the kidney and nourishes the heart, benefits the qi, and promotes the production of body fluid and astringent. Corni fructus tonifies the liver and kidney and astringes the essence. Scorpion and centipede are effective in clearing pain, attacking toxins, and dispersing nodules. *Gekko swinhonis* Seu japonicus dispels wind, settles fright, detoxifies, and disperses nodules. The combination of these drugs can benefit qi and nourish yin, clear heat and detoxify the body, tonify the kidney, and strengthen the spleen. Modern pharmacological research shows that Coicis Semen can exert antitumor effects by inducing tumor cell apoptosis, inhibiting tumor cell division, proliferation, and angiogenesis, hindering tumor cell metastasis, and improving the body's immune function. Astragali Radix contains many chemical components such as astragalus polysaccharides, flavonoids, and saponins, which can play multiple roles, such as significantly antitumor, enhancing cellular immune function, scavenging free radicals in the body, affecting apoptosis, reducing adverse effects of chemotherapy drugs, and inhibiting the vascular system of tumors.

## 5. Conclusion

Stereotactic radiotherapy plus chemotherapy with a TP regimen significantly optimizes the clinical efficacy of the NSCLC treatment, enhances the quality of life of patients, and mitigates the serum CYFRA21-1 and MALAT1 levels, with a high safety profile.

## Figures and Tables

**Figure 1:** Short-term curative effects.

**Figure 2:** Total effective rate in percentage.

**Figure 3:** Quality of life.

**Figure 4:** Overall effectiveness.

**Figure 5:** Comparison of survival curves between two groups.

**Figure 6:** The local recurrence and distant metastasis rate of patients between the two groups.

**Table 1:** Primer sequences of MALAT1/*β*-actin.

	MALAT1	*β*-Actin
F	5′-ATTGAGAAATTTTTCCATCGAGCCTTTTT-3′	5′-CCGACAGGATGCAGAAGGAG-3′
R	5′-TCTGAGTGAAGTGTACTATCCCATCA-3′	5′-AGGATGGAGCCGCCGAT-3′

**Table 2:** Results of short-term curative effects.

Group	Number of cases	CR	PR	SD	PD	Total effective rate (%)
Observation group	40	11	15	9	5	65.00
Control group	40	8	12	12	13	50.00
*χ* ^2^						4.604
*P*						0.032

**Table 3:** Results of quality of life.

Group	Number of cases	Improve	Stable	Reduce	Effective
Observation group	40	17	18	5	87.50
Control group	40	10	20	10	75.00
*χ* ^2^					5.128
*P*					0.024

**Table 4:** Detection results of serum CYFRA21-1 and MALAT1 levels.

Group		CYFRA21-1 (ng/mL)	MALAT1
Observation group	Pretreatment	4.58 ± 0.77	0.48 ± 0.11
	After treatment	2.18 ± 0.59	1.02 ± 0.22

Control group	Pretreatment	4.51 ± 0.65	0.47 ± 0.09
	After treatment	3.01 ± 0.54	0.82 ± 0.18

**Table 5:** Comparison of progression-free survival and total survival between the two groups.

Group	Number of cases	Progression-free survival (months)	Total survival (months)
Observation group	40	10.28 ± 2.01	12.36 ± 2.52
Control group	40	8.17 ± 1.58	10.24 ± 2.11
*t*		5.22	4.079
*P*		<0.001	<0.001

**Table 6:** Comparison of survival rates between the two groups.

Group	Number of cases	Half-year survival rate	1 year survival rate
Observation group	40	34	32
Control group	40	30	22
*χ* ^2^		1.250	5.698
*P*		0.264	0.017

**Table 7:** The local recurrence rate and the distant metastasis rate of patients between the two groups.

Groups	Number of cases	Local recurrence rate	Distant metastasis rate
Observation group	40	2	3
Control group	40	9	10
*χ* ^2^		5.165	4.501
*P*		0.024	0.034

**Table 8:** Investigation results of adverse reactions in patients.

Group	Leukocytopenia	Hemoglobin decrease	Gastrointestinal reaction	Liver function impairment	Renal impairment
Observation group	1 (2.50)	0	0	1 (2.50)	1 (2.50)
Control group	1 (2.50)	2 (5.00)	2 (5.00)	1 (2.50)	4 (10.00)
*χ* ^2^	—	5.128	5.128	—	4.800
*P*	—	0.024	0.024	—	0.029

## Data Availability

The data generated or analyzed during this study are included within the article.
